The article "Long-Term Treatment Outcomes of the Elder Patients with Locally Advanced Thoracic Esophageal Squamous Cell Carcinoma with Definitive Chemoradiotherapy or Radiotherapy" was published in 2022. Journal: Contrast Media Mol Imaging.

# Long-Term Treatment Outcomes of the Elder Patients with Locally Advanced Thoracic Esophageal Squamous Cell Carcinoma with Definitive Chemoradiotherapy or Radiotherapy

**DOI:** 10.1155/2022/3678441

**Published:** 2022-07-16

**Authors:** Junqing Liu, Yishuang Li, Ying Chen, Xue Jiang, Haogang Yu, Senxiang Yan

**Affiliations:** ^1^Department of Radiation Oncology, The First Affiliated Hospital, College of Medicine, Zhejiang University, Hangzhou 310003, China; ^2^Nanchang University Queen Mary School, Nanchang 330000, China

## Abstract

**Background:**

Few randomized trials are available to guide clinical management of elderly patients with esophageal cancer. Therefore, treatment approaches for the elderly are challenging.

**Objective:**

We believe that chemotherapy and radiotherapy are more effective than radiotherapy alone. We envision that chemotherapy is more effective than radiotherapy alone in elderly patients with esophageal cancer.

**Methods:**

Retrospective data of patients aged 70 years and older from 2008 to 2015 at our institution were analyzed. Of 61 eligible patients, 32 received definitive CTR and 29 received RT alone. Progression-free survival (PFS) was 16 months (range, 1–67 months), and the median overall survival was 19 months. Median PFS and OS in the chemoradiotherapy group were 17 months (95% confidence interval (CI), 15.1–24.8 months) and 22 months (95% confidence interval (CI), 20.4–32.7 months), respectively.

**Results:**

The median PFS and OS in the radiotherapy group were 16 months and 16 months, respectively. The OS rates at 1, 2, 3, and 5 years were 82%, 42.6%, 19.7%, and 6.6%, respectively. There was no difference in PFS between CRT and RT, but there was an advantage in OS for CRT. Positive nodules had an effect on PFS and OS.

**Conclusions:**

CRT is effective in elderly patients with nodal invasion of esophageal cancer. Higher radiation doses had an effect on PFS and OS, but there was no difference in PFS and OS between CRT and RT. Therefore, treatment approaches for the elderly are challenging.

## 1. Introduction

Esophageal cancer (EC) is a major health concern worldwide, with nearly 482,300 new cases and 406,800 deaths each year. While esophageal cancer is the eighth most common cancer, with estimated 455,784 new cases, it is the sixth leading cause of cancer death, with 400,156 deaths in 2012. However, in China, esophageal cancer is the fifth most common cancer and the fourth leading cause of cancer death. Esophageal squamous cell carcinoma (ESCC) is the predominant histologic form of esophageal cancer in China, and the common treatment for localized EC is chemotherapy followed by surgery (triple-modality therapy (TMT)) or definitive chemotherapy (dual-modality therapy (BMT)) and palliative or supportive care [1–4]. Some trials of neoadjuvant chemoradiotherapy and definitive surgery in older patients have reported no difference in surgical complications from patients younger than 70 years. At the initial diagnosis, most patients are found to be advanced in older patients. Therefore, it is difficult to have a definitive treatment for elderly patients [5].

The article "Long-Term Treatment Outcomes of the Elder Patients with Locally Advanced Thoracic Esophageal Squamous Cell Carcinoma with Definitive Chemoradiotherapy or Radiotherapy" was published in 2022. Journal: Contrast Media Mol Imaging.

Currently, the number of useful trials on the efficacy of CRT or radiotherapy in elderly patients with locally advanced EC is insufficient, and adequate data on the long-term efficacy of CRT or radiotherapy in such patients are limited [5–8]. According to the NCCN guidelines (2020), we, therefore, conducted a retrospective analysis at a single institution to assess the efficacy of CRT or radiotherapy in EC patients aged ≥70 years and to evaluate the long-term outcome of CRT or radiotherapy in such patients [9–12].

## 2. Methods

### 2.1. Patients

This study was approved by our hospital review board. We retrospectively studied our patient's data for the records of old patients (≥70 years old) with local regionally advanced thoracic esophageal squamous cell carcinoma without operation with curative radiotherapy or chemoradiotherapy between 2008 and 2015. Patients greater than or equal to 70 years old with advanced-stage cancer treated with irradiation or chemoradiotherapy were included. Patients with distant metastasis and patients who received esophageal surgery, second primary carcinoma, and chemotherapy before radiotherapy were excluded. The pathologic diagnosis of esophageal cancer was confirmed by the endoscopic biopsy. Information of the patients from the patient's database included sex, age, tumor stage, pathologic diagnosis, and type of therapy. The patients with esophageal cancers were mainly included in the thoracic region, excluding the tumors in the neck and distal regions or gastroesophageal junction tumors [13–15].

Stage of the most patients was determined by computed tomography; some patients also tested positron emission tomography-computed tomography. The TNM stage was determined by the American Joint Committee on Cancer (7th edition, 2010).

### 2.2. Treatment

Patients included in the research were categorized by the type of therapy. One group accepted for definitive radiotherapy alone, and the other was treated with chemoradiotherapy.

A typical radiotherapy technology included immobilizing the patients in supine position with their arms down. Three-dimensional CT imaging was applied in our study. The three-dimensional conformal technique was applied. The prescription doses for definitive therapy ranged from 50 to 66 Gy. The organs at risk (OAR) were required according to the NCCN Guidelines version [16].

The article "Long-Term Treatment Outcomes of the Elder Patients with Locally Advanced Thoracic Esophageal Squamous Cell Carcinoma with Definitive Chemoradiotherapy or Radiotherapy" was published in 2022. Journal: Contrast Media Mol Imaging.

The chemotherapy regimens were capecitabine (850 mg/m^2^, bid d1-14 q3w), cisplatin (70–80 mg/m^2^), and fluorouracil (700–750 mg/m^2^ civ 96 h, q4 w) according to the patients' KPS score (70–90).

### 2.3. Evaluation and Follow-Up

About 3 months after the treatment for 2 years and every 6 months after 2 years until death or cutoff time after the treatments [17], tumor response was evaluated with physical examination, barium X-ray, and computer tomography according to the new response evaluation criteria in solid tumors: revised RECIST guideline (RECIST 1.1d Update and clarification; from the RECIST criteria) (11–12A, B). The duration of follow-up was 1.5–72 months.

### 2.4. Statistical Analysis

Statistical analysis was used with the chi-squared test for two-proportion comparisons. Overall survival (OS), progress-free survival (PFS), distant metastasis-free survival (DMFS), and local control rate (LCR) were analyzed with the Cox proportional hazard regression model and Kaplan–Meier methodology. Univariate and multivariate analyses were used in the Cox regression model. *P* < 0.05 was considered a statistically significant value. All the analyses were used with SPSS software (SPSS 19.0).

## 3. Results

Outcomes are as follows: at the end of the follow-up time, two patients had lost with an overall follow-up ratio of 96.7%. The median age of the patients was 76 years (range, 70–83 years). The median progression-free survival (PFS) was 16 months (range, 1–67 months) and the median overall survival time was 19 months (range, 1–72 months). Among all the patients, they had chemoradiotherapy treatment with 32 (52.5%) and 29 in the radiotherapy group (47.5%). The median PFS and OS were, respectively, in the chemoradiotherapy group at 17 months (95% confidence interval (CI), 15.1–24.8 months) and 22 months (95% confidence interval (CI), 20.4–32.7 months). The median PFS and OS were, respectively, in the radiotherapy group for 16 months (95% confidence interval (CI), 13.5–26.9 months) and 16 months (95% confidence interval (CI, 10.6–15.3 months). The median PFS in the chemoradiotherapy group is a little longer than that in the radiotherapy group without a significant difference, and the OS in the chemoradiotherapy group is longer than that in radiotherapy without an obvious difference. A total number of 29 patients remained alive with no evidence of disease and 2 patients remained alive but presented with primary recurrence. The 1, 2, 3, and 5-year OS rates were 82%, 42.6%, 19.7%, and 6.6%, respectively. The patients were divided into two classes with negative or positive regional nodes. The 1, 2, 3, and 5-year OS rates with negative regional nodes were 77.1%, 45.7%, 28.6%, and 8.6%, respectively. The 1, 2, 3, and 5-year OS rates with positive regional nodes were 80.8%, 30.8%, 11.5%, and 3.8%, respectively [18, 19].

The article "Long-Term Treatment Outcomes of the Elder Patients with Locally Advanced Thoracic Esophageal Squamous Cell Carcinoma with Definitive Chemoradiotherapy or Radiotherapy" was published in 2022. Journal: Contrast Media Mol Imaging.

Patient features are as follows: the baseline features of the patients are given in Table 1. There was no statistical difference in gender. The patients were in the same stage in T3, but the patients had a different stage in N (N0-2) and radiotherapy dose (Table 1).

Univariate and multivariate analyses are as follows: the factors of PFS and OS that were considered as the significant value in univariate and multivariate analyses are given in Table 2.

The PFS and OS were related to the duration of radiotherapy, local recurrence, and the disease-related death. There was a significant advantage of PFS and OS with multivariate analysis with disease-related death and radiotherapy dose. Kaplan–Meier estimates of PFS and OS are according to the different treatment groups. The PFS and OS were connected with the radiation dose (Figure 1).

The median dose is 60 Gy (range from 50–66 Gy), and the cutoff dose was defined as 54 Gy. The PFS and OS were taken the effect by radiation dose (Figure 2).

The PFS and OS were related to the local recurrence of ESCC (Figure 3).

The PFS and OS were related to ESCC which had a significant difference (Figure 4).

Chemotherapy had no advantage for the PFS and OS with ESCC (Figure 5).

Reason for death is as follows: a total number of 45 patients had attended the follow-up. 26 patients had died of local recurrence and distant metastasis of the primary esophageal carcinoma, and 2 patients had succumbed to radiation complications of pulmonary infection. 5 patients had died of underlying comorbidity, including 2 patients with respiratory failure, 1 patient with pelvic fracture complications, and 1 patient with cerebral infarction. The reason for death in the 9 patients was unknown.

## 4. Discussion

The number of elderly esophageal carcinoma patients is increasing with longevity year by year. So, it is important that elderly patients with their families choose the treatment methods without heavy complications and with improving quality of life. The results of the retrospective study showed that the elderly patients with advanced thoracic esophageal squamous cell carcinoma had no different advantage between chemoradiotherapy and radiotherapy with multivariate analysis, but overall survival rates had been affected by prolonging and interruptions of treatment time of radiotherapy, local recurrence, and cause-specific death with univariate analysis. The prolonged and interrupted treatment time of radiotherapy is a presumed radiobiological explanation for the local regional control as an adverse factor.

The article "Long-Term Treatment Outcomes of the Elder Patients with Locally Advanced Thoracic Esophageal Squamous Cell Carcinoma with Definitive Chemoradiotherapy or Radiotherapy" was published in 2022. Journal: Contrast Media Mol Imaging.

When selecting the therapy method, the quality of life after treatment or during the treatment time is one of the important factors for these elderly patients. Radiotherapy or chemoradiotherapy is a noninvasive treatment that is to be chosen by patients, especially old patients. Hideomi Yamashita reported that the quality of life was superior in the definitive chemoradiotherapy for the clinical stage II-III esophageal carcinoma, although the chemoradiotherapy group was inferior to surgery in survival. Another report also showed CRT improved dysphagia than surgery and CRT had lower complications than surgery in a short time. Now, how to evaluate the survival time of the elderly patients is not clear, and randomized controlled studies of the therapy methods are needed to select treatment options for elderly patients with esophageal cancer.

Most elderly patients with esophageal carcinoma have not accepted the adjuvant chemotherapy after concurrent chemotherapy and radiotherapy or radiotherapy alone. Adjuvant chemotherapy seemed less efficient after surgery with node-negative to improve the overall survival, but adjuvant chemotherapy increased the overall survival with node-positive and margin-positive patients. The JCOG9204 phase III trial showed that there was no advantage in the OS between surgery alone and surgery with adjuvant chemotherapy. Above all, it is unclear whether the elderly patients with definitive treatments should be accepted adjuvant chemotherapy.

Furthermore, the RT dose of ESCC was ambiguous between 50 Gy and more than 60 Gy. Our results showed the high RT dose improved PFS and OS. Some reports demonstrated that a high RT dose of PFS and OS was better than the standard RT dose. Chun-Ru Chien et al. based propensity-score matched analysis had reported a high RT dose as a good prognostic factor. He-San Luo also demonstrated the results. So, it is really important to define the pattern of therapy in elderly ESCC patients. Our data were not enough of patients and needed further randomized controlled trials to confirm the results.

## 5. Conclusions

In our data, the elderly patients' death of locally advanced ESCC is due to the disease-related death. PFS and OS with CCRT were not better than the RT group. A high RT dose was a favorable prognostic factor for the advanced ESCC patients. According to the NCCN guidelines (2020), we, therefore, conducted a retrospective analysis at a single institution to assess the efficacy of CRT or radiotherapy in EC patients aged ≥70 years and to evaluate the long-term outcome of CRT or radiotherapy in such patients. Furthermore, randomized controlled trials are needed to testify our conclusions and confirm the outcomes for higher radiation doses.

The article "Long-Term Treatment Outcomes of the Elder Patients with Locally Advanced Thoracic Esophageal Squamous Cell Carcinoma with Definitive Chemoradiotherapy or Radiotherapy" was published in 2022. Journal: Contrast Media Mol Imaging.

## Figures and Tables

**Figure 1:** PFS and OS comparison chart.

**Figure 2:** Comparison of PFS and OS by radiation dose.

**Figure 3:** Local recurrence of PFS and OS with ESCC.

**Figure 4:** Prefeasibility study vs. OS vs. ESCC.

**Figure 5:** Comparison of chemotherapy on a prefeasibility study.

**Table 1:** Features of the patients.

Features	No. of patients	DM		*P*	Duration of treatment		*P*	LC		*P*
		No (%)	Yes (%)		<6 weeks	≥6 weeks		No (%)	Yes (%)	
		No (%)	No (%)		No (%)	No (%)		No (%)	No (%)	
Gender				0.225			0.924			0.309
Male	52	36 (69.20%)	16 (30.80%)		28 (53.80%)	24 (46.20%)		38 (73.10%)	14 (26.90%)	
Female	9	8 (88.90%)	1 (11.10%)		5 (55.60%)	4 (44.40%)		8 (88.90%)	1 (11.10%)	

cStage				0.311			0.315			0.715
II	35	27 (77.10%)	8 (22.90%)		17 (48.60%)	18 (51.40%)		27 (77.10%)	8 (22.90%)	
III	26	17 (65.40%)	9 (34.60%)		16 (61.50%)	10 (38.50%)		19 (73.10%)	7 (26.90%)	

cN				0.315			0.311			0.715
Yes	26	16 (61.50%)	10 (38.50%)		17 (65.40%)	9 (34.60%)		19 (73.10%)	7 (26.90%)	
No	35	17 (58.6%)	18 (51.40%)		27 (77.10%)	8 (22.90%)		27 (77.10%)	8 (22.90%)	

Method of treatment				0.234			0.5			0.204
CRT	32	21 (65.60%)	11 (34.40%)		16 (50.00%)	16 (50.00%)		22(68.80%)	10 (31.20%)	
RT	29	23 (79.30%)	6 (20.70%)		17 (58.60%)	12 (41.40%)		24(82.80%)	5 (17.20%)	

Dose (Gy)				0.043			0.023			0.858
<54	52	35 (67.30%)	17 (32.70%)		25 (48.10%)	27 (51.90%)		39 (75.50%)	13 (25.00%)	
≤54	9	9 (100%)	0 (0%)		8 (88.90%)	1 (11.10%)		7 (77.80%)	2 (22.20%)	

**Table 2:** Univariate and multivariate Cox regression analyses of PFS and OS.

Parameters	PFS				OS			
	Univariate analysis		Multivariate analysis		Univariate analysis	Multivariate analysis		
	Hazard ratio (95% CI)	*P* value	Hazard ratio (95% CI)	*P* value	Hazard ratio (95% CI)	*P* value	Hazard ratio (95% CI)	*P* value
Type of treatment		0.347				0.319		
CCRT	1 (reference)				1 (reference)			
RT	1.61 (0.85–1.58)				1.45 (0.70–3.03)			

Clinical TNM classification		0.167				0.361		
II	1 (reference)				1 (reference)			
III	0.80 (0.58–1.10)				0.71 (0.34–1.49)			

N stage		0.167				0.361		
N0	1 (reference)				1 (reference)			
N1-2	1.56 (0.83–2.93)				1.41 (0.67–2.98)			

Local recurrence		0.005				0.006		
No	1 (reference)				1 (reference)			
Yes	2.57 (1.33–4.94)				2.83 (1.35–5.91)			

Distant metastasis		0.077				0.537		
No	1 (reference)				1 (reference)			
Yes	1.81 (0.94–3.48)				1.27 (0.60–2.69)			

Duration of treatment		0.058				0.031		
≤6 weeks	1 (reference)				1 (reference)			
>6 weeks	0.54 (0.28–1.02)				0.42 (0.19–0.92)			

Diseases related death		0.001		0.001		0.001		0.000
No	1 (reference)		1 reference		1 (reference)		1 (reference)	
Yes	2.89 (1.51–5.55)		2.89 (1.51–5.55)		3.82 (1.77–8.24)		4.96 (2.19–11.26)	

Dose of irradiation		0.094		0.017		0.071		0.005
≤54 Gy	1 (reference)		1 (reference)		1 (reference)		1 (reference)	
>54 Gy	0.47 (0.19–1.14)		0.33 (0.13–0.82)		0.40 (0.15–1.08)		0.21 (0.07–0.62)	

The article "Long-Term Treatment Outcomes of the Elder Patients with Locally Advanced Thoracic Esophageal Squamous Cell Carcinoma with Definitive Chemoradiotherapy or Radiotherapy" was published in 2022. Journal: Contrast Media Mol Imaging.

## Data Availability

The experimental data used to support the findings of this study are available from the corresponding author upon request.
